The article "Suppression of a single pair of mushroom body output neurons in Drosophila triggers aversive associations" was published in 2017. Journal: FEBS Open Bio.

# Suppression of a single pair of mushroom body output neurons in *Drosophila* triggers aversive associations

**DOI:** 10.1002/2211-5463.12203

**Published:** 2017-02-22

**Authors:** Yutaro Ueoka, Makoto Hiroi, Takashi Abe, Tetsuya Tabata

**Affiliations:** ^1^ Department of Biological SciencesGraduate School of ScienceThe University of TokyoBunkyo‐kuJapan; ^2^ Institute of Molecular and Cellular BiosciencesThe University of TokyoBunkyo‐kuJapan

**Keywords:** dopaminergic, *Drosophila*, MBON, memory acquisition, memory suppression, olfactory aversive memory

## Abstract

Memory includes the processes of acquisition, consolidation and retrieval. In the study of aversive olfactory memory in *Drosophila melanogaster*, flies are first exposed to an odor (conditioned stimulus, CS+) that is associated with an electric shock (unconditioned stimulus, US), then to another odor (CS−) without the US, before allowing the flies to choose to avoid one of the two odors. The center for memory formation is the mushroom body which consists of Kenyon cells (KCs), dopaminergic neurons (DANs) and mushroom body output neurons (MBONs). However, the roles of individual neurons are not fully understood. We focused on the role of a single pair of GABAergic neurons (MBON‐γ1pedc) and found that it could inhibit the effects of DANs, resulting in the suppression of aversive memory acquisition during the CS− odor presentation, but not during the CS+ odor presentation. We propose that MBON‐γ1pedc suppresses the DAN‐dependent effect that can convey the aversive US during the CS− odor presentation, and thereby prevents an insignificant stimulus from becoming an aversive US.

**Abbreviations**
BGAM: blockade of MBON‐γ1pedc‐induced aversive memory
CS: conditioned stimulus
DANs: dopaminergic neurons
ES: electric shock
KCs: Kenyon cells
MB: mushroom body
MBONs: MB output neurons
STM: short‐term memory
US: unconditioned stimulus

Pavlovian classical conditioning, in which the conditioned stimulus (CS) is associated with the unconditioned stimulus (US), serves as a simple model for learning and memory. There are many kinds of stimuli in the environment, and organisms have evolved to select for stimuli that are used as the US in conditioning paradigms, enabling them to survive and thrive. The olfactory aversive memory of *Drosophila melanogaster* serves as a good example of Pavlovian classical conditioning 1, 2, and several distinct stimuli can be used as the US in *Drosophila* 1, 2, 3, 4, 5, 6. However, the mechanisms by which *Drosophila* select the US or tune the threshold for accepting a stimulus as the US remain largely unknown.

The neuropil called the mushroom body (MB) has been extensively studied anatomically 7, 8, 9 and functionally as the center for the olfactory aversive memory 10, 11, 12, 13. The MB consists of ~ 2000 intrinsic neurons called Kenyon cells (KCs), which are the third‐order olfactory neurons in each hemisphere 8. Subsets of KCs sparsely represent odor information 14, 15, 16, 17, and the information is modified by aversive stimuli conveyed by dopaminergic neurons (DANs) upon conditioning 12, 18, 19, 20. The modified information then converges on MB output neurons (MBONs) 9, 21. Cellular identification of MBONs has been an intriguing result from recent studies of brain anatomy 22, 23. It has been revealed that odor information encoded in ~ 2000 KCs converges on only 34 MBONs composed of 21 anatomically distinct cell types 9. This finding permits the study of neuronal mechanisms underlying odor coding and olfactory memory formation in the reduced dimension at the level of fourth‐order olfactory neurons. Specifically, it allows us not only to identify each output neuron at a cellular resolution but also to manipulate the functions of each output neuron using split‐Gal4 drivers 9, 24. We have already started to witness the progress in understanding roles of MBONs in the process of memory formation 9, 21, 22, 23, 25, 26. In addition, the DAN activity has been shown to be dynamically changed by external stimuli or internal physiological states 27, 28, 29, and the output from MBONs is also known to affect the DAN activity 28, suggesting that the circuits consisting of KCs, DANs and MBONs form dynamic neuronal networks including multiple layers of feed forward and feedback regulation.

The article "Suppression of a single pair of mushroom body output neurons in Drosophila triggers aversive associations" was published in 2017. Journal: FEBS Open Bio.

We chose to study the role of MBON‐γ1pedc because it has been reported to play a pivotal role in aversive memory 24, 26 and because a memory trace is detected in its responses to odors associated with electric shocks or activation of DANs 26, 30. In addition, MBON‐γ1pedc reflects internal and physiological states of flies and inhibits activities of other MBONs 26. These results prompted us to explore the possibility that MBON‐γ1pedc plays multiple roles in memory formation, and we found that MBON‐γ1pedc was required for the acquisition of memory. Furthermore, during memory formation, MBON‐γ1pedc suppresses the acquisition of aversive memory for CS− but not for CS+.

## Materials and Methods

### Fly strains

All flies were raised on standard cornmeal‐agar food at 25 °C. Flies of either sex were used in this study. *CS10* (*w1118* backcrossed with *Canton‐S* for 10 generations) was used as a control strain in this study. Generation and basic characterization of the split‐Gal4 drivers (*MB112C, MB060B, MB504B*, and *MB438B*) are described in 9, and these drivers were kindly provided by the Rubin lab. Further information and line generation is available at https://www.janelia.org/split-gal4. *TH‐Gal4* 31 was obtained from M. Heisenberg. *pJFRC99‐20XUAS‐IVS‐Syn21‐Shibire‐ts1‐p10* in *VK00005* 32 was obtained from the HHMI Janelia Farm Fly Facility. *UAS‐mCherry.NLS* (http://flybase.org/reports/FBrf0218019.html), *UAS‐dTrpA1 in attP16* 33, *UAS‐mCD8::GFP* 34, *UAS‐mCD8::RFP in attP18 LexAop‐mCD8::GFP in su(Hw)attP8*,* R83A12‐Gal4 in attP2* and *R12G04‐LexA in attP40* were obtained from Bloomington (#38425, #26263, #5130, #32229, #40348, #52448). [Correction added after online publication on 22 March 2017: corrections made to fly strain information].

The article "Suppression of a single pair of mushroom body output neurons in Drosophila triggers aversive associations" was published in 2017. Journal: FEBS Open Bio.

### Setting for behavioral experiments

Groups of ~ 50 flies (2–5 days old) raised under a 12 hr:12 hr light–dark cycle were used for one trial in behavioral experiments. Before behavior experiments, flies were kept in vials with Kimwipes soaked with sucrose solution. The training and test apparatus were the same as described previously 2, and protocols were slightly modified. Flies were exposed to 60 s of a CS+ odor (MCH or OCT) with 12 90 V electric shocks at a 5 s interstimulus interval, then 30 s of clean air, followed by the CS− odor (OCT or MCH) without electric shocks. After the training stage, flies were allowed to select the CS+ odor or the CS− odor in a T‐maze at test stage. Odors were in a glass ‘odor cup’ (8 mm in diameter for OCT and 10 mm for MCH) sitting in the middle of an odor stream. The flow velocities of air or odors were 0.75 L·min^−1^ in each stage.

### Temperature shifting

To shift temperature between the permissive temperature (22 °C) and the restrictive temperature (33 °C), we used two climate boxes set to 22 °C or 33 °C, and all of the training tubes and T‐mazes were preheated and fixed at the indicated temperatures. Temperature shifts were performed immediately. After the transfer, flies were left in a tube with airflow at the indicated temperature.

### Temperature shifting between training and test

Flies were preheated at 33 °C for 30 min and then trained and tested at 33 °C (Fig. 1D). Flies were trained and tested at 22 °C (Fig. 1E). Flies were preheated at 33 °C for 30 min, trained at 33 °C, and then transferred to 22 °C and tested at 22 °C (Figs 1F, 4C). [Corrections added after online publication on 22 March 2017: figure citations altered]. Flies were trained at 22 °C and then transferred to 33 °C and tested at 33 °C (Fig. 1G).

**Figure 1:** MBON‐γ1pedc is required for both acquisition and retrieval of STM. (A) Olfactory aversive memory assay scheme. At the training/acquisition stage, one odor (CS+) is delivered to flies with 12 electric shocks, and another odor (CS−) is delivered without a shock for 1 min. After that, flies are allowed to choose between the CS+ odor and CS− odor at the test stage. (B–C) MB112C split‐Gal4 expressing UAS‐mCD8::GFP and UAS‐nls::mCherry labeled single pair of MBON‐γ1pedc. Scale bars, 50 μm. (D) Blocking synaptic outputs from MBON‐γ1pedc during the training and test stages impaired short‐term memory (STM) (ANOVA,* n* = 8, 9, 7). Flies were preheated at the restrictive temperature (33 °C) before training for 30 min, followed by training and testing at 33 °C. (E) Flies showed no deficit in STM at the permissive temperature (22 °C). Flies expressing Shi^ts^ in MBON‐γ1pedc showed no significant memory deficits compared to the relevant Gal4 or UAS‐Shi^ts^ controls (Kruskal–Wallis, *n* = 7, 7, 7). Flies were trained and tested at 22 °C. (F) Blocking synaptic outputs from MBON‐γ1pedc at the training stage impaired STM (ANOVA,* n* = 8, 8, 8). Flies were preheated at 33 °C before training for 30 min, followed by training at 33 °C. Immediately after the training, flies were transferred to 22 °C and tested at 22 °C. (G) Blocking synaptic outputs from MBON‐γ1pedc at the test stage impaired STM (ANOVA,* n* = 7, 6, 6). Flies were trained at 22 °C, followed by a transfer to 33 °C and testing at 33 °C. (D‐G) All bar graphs show the mean ± SEM, and dots show individual trials. *: *P* < 0.05, **: *P* < 0.01, ***: *P* < 0.001, n.s.: *P* > 0.05.

The article "Suppression of a single pair of mushroom body output neurons in Drosophila triggers aversive associations" was published in 2017. Journal: FEBS Open Bio.

### Temperature shift during CS+ and CS− presentation

Flies were trained with the CS+ presentation at 22 °C and immediately transferred to 33 °C, followed by 2 min air flow, and the CS− was presented at 33 °C, then immediately retransferred to 22 °C, followed by 2 min air flow and testing at 22 °C (Figs 2A, 4D, 5B). These tests used the same protocol as in Figs 2A, 4D and 5B with only the timing of electric shocks changed, thus switching the CS+ and CS− (Figs 2B, 4E, 5C). [Corrections added after online publication on 22 March 2017: figure citations altered]. Flies were trained with the CS+ presentation at 22 °C and immediately transferred to 33 °C, followed by 3 min air flow at 33 °C, and they were then immediately retransferred to 22 °C, followed by 2 min air flow, the CS− presentation at 22 °C and testing at 22 °C (Fig. 2C). Flies were preheated at 33 °C for 30 min, trained with the CS− presentation at 33 °C, and then immediately transferred to 22 °C, followed by 2 min air flow and the CS+ presentation at 22 °C, with testing at 22 °C (Fig. 2D).

**Figure 2:** Blockade of MBON‐γ1pedc during the presentation of CS‐ causes memory deficits. (A) Blocking synaptic outputs from MBON‐γ1pedc during the CS− presentation impaired short‐term memory (STM) (ANOVA,* n* = 12, 12, 12). (B) Blocking synaptic outputs from MBON‐γ1pedc during the CS+ presentation did not impair STM (Kruskal–Wallis, *n* = 6, 6, 6). (C) Blocking synaptic outputs from MBON‐γ1pedc immediately after the CS+ presentation did not impair STM (ANOVA,* n* = 8, 8, 8). (D) Blocking synaptic outputs from MBON‐γ1pedc during the CS− presentation impaired STM (ANOVA,* n* = 11, 12, 11). This is the sequential control to A. (A–D) All bar graphs show the mean ± SEM, and dots show individual trials. *: *P* < 0.05, **: *P* < 0.01, n.s.: *P* > 0.05.

The article "Suppression of a single pair of mushroom body output neurons in Drosophila triggers aversive associations" was published in 2017. Journal: FEBS Open Bio.

### Blockade of MBON‐γ1pedc‐induced aversive memory (BGAM) training and test

Flies were exposed to odor 1 for 60 s at 22 °C and immediately transferred to 33 °C, followed by 2 min air flow, exposure to odor 2 for 60 s at 33 °C, and then immediate retransfer to 22 °C, followed by 2 min air flow and testing at 22 °C (Figs 3B, 4F, 5A and 6B,C).

**Figure 3:** Flies acquired the aversive memory for odors sensed without output from MBON‐γ1pedc. (A) Blockade of MBON‐γ1pedc‐induced aversive memory (BGAM) scheme. At the training/acquisition stage, one odor is delivered to flies at the permissive temperature for 1 min followed by temperature shifting to the restrictive temperature, and another odor is delivered at the restrictive temperature for 1 min. Subsequently, the flies are allowed to choose between the odors at the test stage. (B) Blocking synaptic outputs from MBON‐γ1pedc during odor presentation caused aversive STM, as compared to controls (ANOVA,* n* = 7,8,7). The performance index in this figure was calculated for odor 2, and the positive index indicates that flies avoid odor 2 over odor 1. (C) Single odor presentation during the blockade of MBON‐γ1pedc caused significant aversive STM, as compared to control strains (ANOVA,* n* = 11, 12, 11). The Performance Index in this figure was calculated for the odor presented at the restrictive temperature, and the positive index indicates that flies avoid the odor over another control odor that was not presented during training. (B–C) All bar graphs are mean ± SEM, and dots represent individual trials. **: *P* < 0.01.

**Figure 4:** R83A12 driver also induced STM acquisition impairment and BGAM formation. (A, A’) *MB112C‐splitGal4* and *R12G04‐LexA* expressed mCD8::RFP and mCD8::GFP, respectively. Both drivers label MBON‐γ1pedc. Scale bars: 50 μm. (B, B’) *R83A12‐Gal4* and *R12G04‐LexA* expressed mCD8::RFP and mCD8::GFP, respectively. Both drivers label MBON‐γ1pedc. Scale bars: 50 μm. (C) Blocking synaptic outputs from R83A12‐positive neurons at the training stage impaired STM (ANOVA,* n* = 11, 11, 10). The flies were preheated at 33 °C before training for 30 min at 33 °C. Immediately after the training, the flies were transferred to 22 °C and tested at 22 °C. (D) Blocking synaptic outputs from R83A12‐positive neurons during the CS‐ presentation impaired STM (ANOVA,* n* = 7, 7, 6). (E) Blocking synaptic outputs from R83A12‐positive neurons during the CS+ presentation did not impair STM (ANOVA,* n* = 7, 8, 7). (F) Blocking synaptic outputs from R83A12‐positive neurons during odor presentation caused aversive STM, as compared to controls (ANOVA,* n* = 8, 9, 7). The Performance Index in this figure was calculated for odor 2, and the positive index indicates that flies avoid odor 2 over odor 1. (C–F) All bar graphs are mean ± SEM, and dots represent individual trials. *: *P* < 0.05, **: *P* < 0.01, n.s.: *P* > 0.05.

The article "Suppression of a single pair of mushroom body output neurons in Drosophila triggers aversive associations" was published in 2017. Journal: FEBS Open Bio.

**Figure 5:** BGAM is acquired through DANs, and blocking DANs rescued the memory deficits caused by BGAM. (A) BGAM was completely diminished by blocking the synaptic output from DANs during the odor 2 presentation (Kruskal–Wallis, *n* = 8, 8, 10, 8). Blocking DANs did not cause any difference as compared to other controls. (B) Blocking synaptic outputs from DANs during the CS− presentation rescued the memory impairment caused by BGAM (Kruskal–Wallis, *n* = 9, 8, 9, 8). (C) Blocking synaptic outputs from DANs during the CS+ presentation impaired STM, regardless of the MBON‐γ1pedc output (ANOVA,* n* = 9, 10, 10, 7). (D) Activating MBON‐γ1pedc during CS+ presentation did not impair STM (ANOVA,* n* = 7, 7, 8). (A–D) All bar graphs are mean ± SEM, and dots represent individual trials. *: *P* < 0.05, ***: *P* < 0.001, n.s.: *P* > 0.05.

**Figure 6:** Through subsets of DANs, flies acquire BGAM. (A) Blockade of MBON‐γ1pedc‐induced aversive memory (BGAM) scheme. (B) Blocking synaptic outputs from a subset of DANs during odor presentation affected BGAM (ANOVA followed by Dunnett's test comparing with *MB112C/UAS‐Shi* ^*ts*^, *n* = 8–10). (C) Blocking synaptic outputs from PPL1‐γ1pedc during odor presentation did not affect BGAM (ANOVA followed by Dunnett's test comparing with *MB112C/UAS‐Shi* ^*ts*^, *n* = 7, 7, 8, 8). (D) Expression patterns of specific drivers. The gray scale represents subjectively determined intensities of termini in the MB. Partially modified from 39, 40. (B, C) All bar graphs are mean ± SEM, and dots represent individual trials. **: *P* < 0.01, ***: *P* < 0.001, n.s.: *P* > 0.05.

### Test stage

Flies were loaded into the T‐maze and allowed to choose between MCH and OCT for 1.5 min. Performance index was calculated as the number of flies avoiding the CS+ odors (or odors presented at 33 °C for BGAM) minus the number of flies in the other side, divided by the total number of flies. Flies were reciprocally trained with MCH or OCT. Control odors (OCT or MCH) were also presented, and two performance indices each were calculated for MCH and for OCT. The final performance index was calculated by averaging the two performance indices for MCH and for OCT.

The article "Suppression of a single pair of mushroom body output neurons in Drosophila triggers aversive associations" was published in 2017. Journal: FEBS Open Bio.

### Confocal imaging

Flies were dissected in cold phosphate‐buffered saline (PBS) solution and fixed in PBT (PBS containing 0.3% TritonX‐100) with 4% formaldehyde for 30 min at room temperature. After PBT washing, PBT was replaced with PBS, and brains were placed between a glass slide and a cover glass with medium (VECTASHIELD Mounting Medium, Vector Laboratories, Burlingame, CA, USA). Images were captured on a LSM 710 confocal microscope (Carl‐Zeiss, Jena, Germany) and brightness was lineally processed using fiji software (http://fiji.sc/Fiji).

### Statistical analysis

We performed statistical analyses using prism 6 (GraphPad, La Jolla, CA, USA). All behavior data were tested for normality. If all of the number of the data was larger than 7, we performed the D'Agostino & Pearson's omnibus normality test. If the smallest number of the data was 7 or 6, we performed the Shapiro–Wilk normality test or the Kalmogorov–Smirnov normality test, respectively. All data passing the normality tests also passed homogeneity of variance (Bartlett's test). Data showing Gaussian distribution were analyzed using one‐way ANOVA followed by Tukey's multiple comparisons test, except for Fig. 6B,C. Data in Fig. 6B,C were analyzed using one‐way ANOVA followed by Dunnett's test compared with MB112C/UAS‐Shi^ts^. For non‐Gaussian distributed data, Kruskall–Wallis test was performed followed by Dunn's multiple comparisons test. Statistical significance was defined as *P* < 0.05. All bar graphs were created in prism 6. All the statistical analysis data is described in Table 1. In bar graphs, asterisks or n.s. indicate statistical significance; with multiple comparisons some bars are grouped according to *P*‐values, with the largest *P*‐value within the group indicated.

**Table 1:** Statistical analysis

Figure	Normality test	Multiple comparisons test	Combination	Summary	Adjusted *P* value
1D	Shapiro–Wilk normality test	ANOVA followed by Tukey's multiple comparisons test	*Shi/+ vs. MBON‐γ1pedc/+*	ns	0.7134
			*Shi/+ vs. MBON‐γ1pedc>Shi*	***	< 0.0001
			*MBON‐γ1pedc/+ vs. MBON‐γ1pedc>Shi*	***	0.0003
1E	Shapiro–Wilk normality test	Kruskal–Wallis test followed by Dunn's multiple comparisons test	*Shi/+ vs. MBON‐γ1pedc/+*	ns	> 0.9999
			*Shi/+ vs. MBON‐γ1pedc>Shi*	ns	0.4292
			*MBON‐γ1pedc/+ vs. MBON‐γ1pedc>Shi*	ns	> 0.9999
1F	D'Agostino & Pearson omnibus normality test	ANOVA followed by Tukey's multiple comparisons test	*Shi/+ vs. MBON‐γ1pedc/+*	ns	0.6139
			*Shi/+ vs. MBON‐γ1pedc>Shi*	**	0.0018
			*MBON‐γ1pedc/+ vs. MBON‐γ1pedc>Shi*	*	0.0163
1G	Kalmogorov–Smirnov normality test	ANOVA followed by Tukey's multiple comparisons test	*Shi/+ vs. MBON‐γ1pedc/+*	ns	0.9976
			*Shi/+ vs. MBON‐γ1pedc>Shi*	**	0.0015
			*MBON‐γ1pedc/+ vs. MBON‐γ1pedc>Shi*	**	0.0018
2A	D'Agostino & Pearson omnibus normality test	ANOVA followed by Tukey's multiple comparisons test	*Shi/+ vs. MBON‐γ1pedc/+*	ns	0.7175
			*Shi/+ vs. MBON‐γ1pedc>Shi*	**	0.0058
			*MBON‐γ1pedc/+ vs. MBON‐γ1pedc>Shi*	*	0.0398
2B	Kalmogorov–Smirnov normality test	Kruskal–Wallis test followed by Dunn's multiple comparisons test	*Shi/+ vs. MBON‐γ1pedc/+*	ns	0.4329
			*Shi/+ vs. MBON‐γ1pedc>Shi*	ns	> 0.9999
			*MBON‐γ1pedc/+ vs. MBON‐γ1pedc>Shi*	ns	0.9912
2C	D'Agostino & Pearson omnibus normality test	ANOVA followed by Tukey's multiple comparisons test	*Shi/+ vs. MBON‐γ1pedc/+*	ns	0.3798
			*Shi/+ vs. MBON‐γ1pedc>Shi*	ns	0.6398
			*MBON‐γ1pedc/+ vs. MBON‐γ1pedc>Shi*	ns	0.8956
2D	D'Agostino & Pearson omnibus normality test	ANOVA followed by Tukey's multiple comparisons test	*Shi/+ vs. MBON‐γ1pedc/+*	ns	0.9623
			*Shi/+ vs. MBON‐γ1pedc>Shi*	**	0.0049
			*MBON‐γ1pedc/+ vs. MBON‐γ1pedc>Shi*	**	0.008
3B	Shapiro–Wilk normality test	ANOVA followed by Tukey's multiple comparisons test	*Shi/+ vs. MBON‐γ1pedc/+*	ns	0.6803
			*Shi/+ vs. MBON‐γ1pedc>Shi*	***	0.0004
			*MBON‐γ1pedc/+ vs. MBON‐γ1pedc>Shi*	**	0.0018
3C	D'Agostino & Pearson omnibus normality test	ANOVA followed by Tukey's multiple comparisons test	*Shi/+ vs. MBON‐γ1pedc/+*	ns	0.1224
			*Shi/+ vs. MBON‐γ1pedc>Shi*	**	0.0016
			*MBON‐γ1pedc/+ vs. MBON‐γ1pedc>Shi*	***	< 0.0001
4C	D'Agostino & Pearson omnibus normality test	ANOVA followed by Tukey's multiple comparisons test	Shi/+ vs. R83A12/+	ns	0.4911
			Shi/+ vs. R83A12 > Shi	*	0.0317
			R83A12/+ vs. R83A12 > Shi	**	0.0019
4D	Kalmogorov–Smirnov normality test	ANOVA followed by Tukey's multiple comparisons test	Shi/+ vs. R83A12/+	ns	0.9334
			Shi/+ vs. R83A12 > Shi	**	0.0032
			R83A12/+ vs. R83A12 > Shi	**	0.0066
4E	Shapiro–Wilk normality test	ANOVA followed by Tukey's multiple comparisons test	Shi/+ vs. R83A12/+	ns	0.458
			Shi/+ vs. R83A12 > Shi	ns	0.7599
			R83A12/+ vs. R83A12 > Shi	ns	0.1518
4F	Shapiro–Wilk normality test	ANOVA followed by Tukey's multiple comparisons test	Shi/+ vs. R83A12/+	ns	0.9007
			Shi/+ vs. R83A12 > Shi	*	0.0284
			R83A12/+ vs. R83A12 > Shi	**	0.0095
5A	D'Agostino & Pearson omnibus normality test	Kruskal–Wallis test followed by Dunn's multiple comparisons test	*TH>Shi vs. MBON‐γ1pedc/TH*	ns	> 0.9999
			*TH>Shi vs. MBON‐γ1pedc,TH>Shi*	ns	> 0.9999
			*TH>Shi vs. MBON‐γ1pedc>Shi*	***	0.0003
			*MBON‐γ1pedc/TH vs. MBON‐γ1pedc,TH>Shi*	ns	> 0.9999
			*MBON‐γ1pedc/TH vs. MBON‐γ1pedc>Shi*	*	0.0199
			*MBON‐γ1pedc,TH>Shi vs. MBON‐γ1pedc>Shi*	**	0.0036
5B	D'Agostino & Pearson omnibus normality test	Kruskal–Wallis test followed by Dunn's multiple comparisons test	*TH>Shi vs. MBON‐γ1pedc/TH*	ns	> 0.9999
			*TH>Shi vs. MBON‐γ1pedc,TH>Shi*	ns	> 0.9999
			*TH>Shi vs. MBON‐γ1pedc>Shi*	**	0.0014
			*MBON‐γ1pedc/TH vs. MBON‐γ1pedc,TH>Shi*	ns	> 0.9999
			*MBON‐γ1pedc/TH vs. MBON‐γ1pedc>Shi*	**	0.0035
			*MBON‐γ1pedc,TH>Shi vs. MBON‐γ1pedc>Shi*	*	0.0105
5C	D'Agostino & Pearson omnibus normality test	ANOVA followed by Tukey's multiple comparisons test	*TH>Shi vs. MBON‐γ1pedc/TH*	***	< 0.0001
			*TH>Shi vs. MBON‐γ1pedc,TH>Shi*	ns	0.7708
			*TH>Shi vs. MBON‐γ1pedc>Shi*	***	< 0.0001
			*MBON‐γ1pedc/TH vs. MBON‐γ1pedc,TH>Shi*	***	0.0003
			*MBON‐γ1pedc/TH vs. MBON‐γ1pedc>Shi*	ns	0.9355
			*MBON‐γ1pedc,TH>Shi vs. MBON‐γ1pedc>Shi*	***	0.0002
5D	Shapiro‐Wilk normality test	ANOVA followed by Tukey's multiple comparisons test	*dTrpA1/+ vs. MBON‐γ1pedc/+*	ns	0.9969
			*dTrpA1/+ vs. MBON‐γ1pedcC>dTrpA1*	ns	0.6142
			*MBON‐γ1pedc/+ vs. MBON‐γ1pedc>dTrpA1*	ns	0.6614
6B	D'Agostino & Pearson omnibus normality test	ANOVA followed by Dunnett's multiple comparisons test	*MBON‐γ1pedc>Shi vs. MBON‐γ1pedc,TH>Shi*	***	< 0.0001
			*MBON‐γ1pedc>Shi vs. MB060B>Shi*	***	0.0007
			*MBON‐γ1pedc>Shi vs. MBON‐γ1pedc,MB060B>Shi*	ns	0.7626
			*MBON‐γ1pedc>Shi vs. MB504B>Shi*	***	< 0.0001
			*MBON‐γ1pedc>Shi vs. MBON‐γ1pedc,MB504B>Shi*	***	0.0002
6C	Shapiro–Wilk normality test	ANOVA followed by Dunnett's multiple comparisons test	*MBON‐γ1pedc>Shi vs. MB438B>Shi*	**	0.0033
			*MBON‐γ1pedc>Shi vs. MB438B/MBON‐γ1pedc*	**	0.0027
			*MBON‐γ1pedc>Shi vs. MBON‐γ1pedc,MB438B>Shi*	ns	0.3367

Statistical analyses of the behavioral experiments are summarized. The figure number (first column), the types of normality test (second column), the types of multiple comparisons test (third column), the data for comparison (fourth column), the significance symbol; *indicates *P* < 0.05, **indicates *P* < 0.01, ***indicates *P* < 0.001 and ns indicates *P* > 0.05 (fifth column) and the specific *P* value (sixth column) are indicated. See Materials and methods for details about the type of tests. [Correction added after online publication on 8 March 2017: data for 5D added]. [Corrections added after online publication on 22 March 2017: **** changed to ***].

The article "Suppression of a single pair of mushroom body output neurons in Drosophila triggers aversive associations" was published in 2017. Journal: FEBS Open Bio.

## Results

### MBON‐γ1pedc is required for both acquisition and retrieval of aversive short‐term memory

We first examined the role of MBON‐γ1pedc in 2 min short‐term memory (STM). We used a MBON‐γ1pedc specific split‐Gal4 driver, MB112C (Fig. 1B,C) 9, 24 to express a temperature‐sensitive dominant‐negative form of dynamin, Shi^ts^ 32, 35 and block output from MBON‐γ1pedc. Flies were exposed to an odor, 4‐methylcyclohexanol (MCH) or 3‐octanol (OCT), paired with 12 electric shocks for 1 min (CS+), followed by OCT (or MCH) without electric shocks for 1 min (CS−) (Fig. 1A). Two minutes later, flies were allowed to select one of the two odors to avoid. Flies were trained and tested at a restrictive temperature (33 °C) (Fig. 1D) or at a permissive temperature (22 °C) (Fig. 1E) throughout the experiments. Blocking MBON‐γ1pedc severely impaired STM (Fig. 1D), demonstrating that MBON‐γ1pedc output is indispensable for STM, as has been reported for 2 h memory 24. To clarify whether this STM deficit was caused by impairment of memory acquisition or retrieval, we blocked output from MBON‐γ1pedc during the acquisition stage or the retrieval stage. STM was impaired by blockade of MBON‐γ1pedc either during the training stage (Fig. 1F) or during the test stage (Fig. 1G). These results suggest that MBON‐γ1pedc is required for aversive memory acquisition in addition to aversive memory retrieval 26.

### MBON‐γ1pedc synaptic output is necessary to inhibit aversive memory acquisition for CS−

For further analysis of MBON‐γ1pedc in memory acquisition, we blocked MBON‐γ1pedc separately during the CS+ or CS− presentation. Interestingly, blocking MBON‐γ1pedc during the CS− presentation impaired memory significantly (Fig. 2A), whereas blocking MBON‐γ1pedc during the CS+ presentation (Fig. 2B) or immediately after the CS+ presentation (Fig. 2C) did not cause the memory deficit. The memory deficit was observed regardless of the sequence of odor presentation; flies trained with the CS− presentation at 33 °C followed by CS+ presentation at 22 °C also showed the memory deficit (Fig. 2D). These results indicate that aversive memory acquisition requires MBON‐γ1pedc output during the presentation of the CS− odor (Fig. 2A,D). Blockade of MBON‐γ1pedc during the CS− presentation may interfere with aversive memory acquired during the CS+ presentation.

Considering the possibility that blocking MBON‐γ1pedc during the CS− presentation alone may forms an aversive memory for the CS− odor, and competition of the aversive memory between the CS+ odor and the CS− odor might cause the memory deficit, flies were exposed to two odors in sequence, followed by the test stage. One odor was presented at the permissive temperature, and the other was at the restrictive temperature to block MBON‐γ1pedc (Fig. 3A). We found that flies formed aversive memory toward the odors presented without synaptic output from MBON‐γ1pedc (Fig. 3B). We named this BGAM, blockade of MBON‐γ1pedc‐induced aversive memory. In BGAM acquisition, a control odor is presented before the temperature shift. We investigated the possibility that some type of memory could be formed for the control odor by temperature shifting immediately after the presentation of the odor, since the timing‐dependent behavioral plasticity was reported 36. To test this possibility, only a single odor was presented at the restricted temperature in the training session, and the control odor was not presented. As a result, BGAM was also observed in the training session, regardless of the presentation of the control odor at the permissive temperature (Fig. 3C). These results indicate that the memory deficit evoked by blocking MBON‐γ1pedc at the acquisition stage (Fig. 1F) is caused at least in part by competition between the aversive memory for CS+ and the BGAM for CS−. Thus, output from MBON‐γ1pedc is necessary to prevent the aversive memory for CS−.

The article "Suppression of a single pair of mushroom body output neurons in Drosophila triggers aversive associations" was published in 2017. Journal: FEBS Open Bio.

### MBON‐γ1pedc, but not the other neurons that could also be labeled by the MB112C driver, is responsible for aversive memory acquisition and BGAM

In the above experiments, MB112C was used as the specific driver to label MBON‐γ1pedc. Although MBON‐γ1pedc seemed to be the only neurons labeled by the MB112C driver, according to the confocal images, a few neurons may be labeled by MB112C (Fig. 4A,A’). To test if MBON‐γ1pedc, but not the other neurons, is responsible for aversive memory acquisition and BGAM, R83A12 was used as another driver to examine the role of MBON‐γ1pedc (Fig. 4B,B’). The blockade of the R83A12‐positive neurons by Shi^ts^ impaired STM acquisition (Fig. 4C). Output from the R83A12‐positive neurons was necessary during the CS− presentation (Fig. 4D), but not during the CS+ presentation (Fig. 4E). Furthermore, BGAM was also observed by blocking the R83A12‐positive neurons during odor presentation (Fig. 4F). These results indicate that the neurons responsible for STM acquisition and BGAM formation were likely to be MBON‐γ1pedc, but not the other neurons that could potentially be labeled by the drivers.

### DANs are required for the BGAM acquisition

MBONs and DANs constitute microcircuits 7, 9, and DANs transmit various kinds of aversive information 12, 37, 38, 39. Thus, we tested whether DANs are involved in the BGAM acquisition. To label DANs, we used tyrosine‐hydroxylase (TH) Gal4 (TH‐Gal4) 31, which is thought to label most DANs that convey aversive information 18, 40. Flies lacking synaptic outputs from both MBON‐γ1pedc and DANs showed severe impairment of the BGAM (Fig. 5A), suggesting that the BGAM is made only when MBON‐γ1pedc is inactive and DANs are active. Activation of DANs during the CS− presentation might be the cause of the memory deficit observed when blocking MBON‐γ1pedc during the acquisition stage (Fig. 1F). To test this possibility, we expressed Shi^ts^ in MBON‐γ1pedc and DANs, and performed the same protocol as in Fig. 2A,B. Blocking MBON‐γ1pedc alone during the CS− presentation impaired memory, whereas blocking both MBON‐γ1pedc and DANs during the CS− presentation did not produce any memory impairments (Fig. 5B), indicating that blocking MBON‐γ1pedc during the CS− presentation caused memory deficits via the output of DANs. On the other hand, blocking DANs during the CS+ presentation caused memory deficits with or without the blockade of MBON‐γ1pedc (Fig. 5C). Blocking MBON‐γ1pedc during the CS+ presentation did not cause any significant effects on memory compared to the control Gal4 strain, nor did it rescue memory deficits caused by the blockade of DANs. Assuming that DANs activation is necessary at the CS+ presentation and MBON‐γ1pedc inhibits the effect of DANs, we investigated whether the activation of MBON‐γ1pedc at the CS+ presentation impaired the STM. To activate MBON‐γ1pedc artificially, dTrpA1, a temperature‐sensitive cation channel 33, was expressed by using the MB112C driver. Neurons expressing dTrpA1 are transiently activated at the restrictive temperature (33 °C), and not at the permissive temperature (22 °C). The flies were transferred to the restrictive temperature and immediately the CS+ odor and ESs were presented for 1 min. The flies were then re‐transferred to the permissive temperature, exposed to the CS− odor and tested. This manipulation of MBON‐γ1pedc did not impair the aversive STM significantly (Fig. 5D). The dTrpA1 inducing the artificial activation of MBON‐γ1pedc might be too weak to suppress the effect of DANs induced by ESs sufficiently. Thus, MBON‐γ1pedc might suppress the weak effect of DANs.

The article "Suppression of a single pair of mushroom body output neurons in Drosophila triggers aversive associations" was published in 2017. Journal: FEBS Open Bio.

### DANs are effectively downstream of MBON‐γ1pedc in the acquisition of the memory

Taken together, in classical conditioning, the output of DANs is ineffective in the CS− presentation and is required during the CS+ presentation, whereas the MBON‐γ1pedc output is required during the CS− presentation, but not during the CS+ presentation. In addition, aversive memory induced by the output of DANs in classical conditioning was not affected by blocking MBON‐γ1pedc during CS+ presentation (Fig. 5C), whereas BGAM induced by blocking MBON‐γ1pedc was affected by blocking DANs (Fig. 5A). Thus, DANs are effectively downstream of MBON‐γ1pedc in the aversive memory acquisition stage. In addition, MBON‐γ1pedc and DANs negatively modify each other's functions, since DANs attenuate input from KCs to MBON‐γ1pedc 30, and this study suggests that MBON‐γ1pedc inhibits the functions of DANs.

For further dissection of the involvement of DANs in BGAM, we used a panel of split‐Gal4 drivers 9 and manipulated subsets of TH‐Gal4 positive neurons. We first used drivers to label a large population of TH‐Gal4 positive neurons in combination with MB112C to block the subsets of DANs and MBON‐γ1pedc (Fig. 6B). Compared to the MBON‐γ1pedc blocked flies, flies without synaptic output from MBON‐γ1pedc and TH‐ or MB504B‐positive DANs showed significantly lower BGAM. Blockade of DANs labeled using MB060B did not cause a significant decrease in BGAM. These results indicate that DANs labeled by TH or MB504B, but not by MB060B, are important for BGAM formation. Importantly, MB060B and MB504B label similar subsets of DANs, but only MB504B labels PPL1‐γ1pedc DANs. We next used the MB438B split‐Gal4 driver to manipulate PPL1‐γ1pedc DANs and tested if the BGAM was impaired by blocking PPL1‐γ1pedc DANs and MBON‐γ1pedc, and found that inactivation of PPL1‐γ1pedc DANs did not impair the BGAM (Fig. 6C). Taking into account that MB504B positive neurons are sufficient to suppress the BGAM, a combination of the PPL1‐γ1pedc, ‐γ2α’1, ‐α’2α2 and ‐α3 DANs or all of them are required for BGAM. Since the combination of DANs labeled by MB060B, which does not label PPL1‐γ1pedc DANs, or MB438B, which does not label PPL1‐γ2α’1 DANs, is not sufficient to suppress the BGAM, the PPL1‐γ1pedc DANs and PPL1‐γ2α’1 DANs are necessary for the BGAM. No drivers labeling the combination of PPL1‐γ1pedc, ‐γ2α’1 and ‐α3 DANs or the combination of PPL1‐γ1pedc, ‐γ2α’1 and ‐α’2α2 DANs are available, and thus the necessities for the PPL1‐α’2α2 and ‐α3 DANs are unclear.

Taken together, the BGAM is acquired through a combination of PPL1‐DANs labeled by MB504B, which is consistent with the notion that some DANs function coordinately 19, 27, 28, 40, 41. Their anatomical connectivity also suggests the possibility that MBON‐γ1pedc modify the effects of some DANs projecting to α/β lobes 9, 42.

## Discussion

We have shown that the synaptic output from MBON‐γ1pedc is required for suppressing aversive memory acquisition without electric shocks and that in the classical olfactory conditioning procedure with electric shocks as the US, MBON‐γ1pedc must be active during the CS− presentation, whereas DANs must be active during the CS+ presentation. Given that the memory is formed regardless of the activity of MBON‐γ1pedc during the CS+ presentation and that DANs are required for BGAM, DANs are functionally downstream of MBON‐γ1pedc in this context. Among the population of DANs, BGAM required PPL1‐DANs, which are thought to convey punitive information and cause aversive memory in concert 40, 41. In aversive olfactory memory, electric shocks as the US can be replaced by artificial activation of PPL1‐DANs 18, 19, 43, indicating that DAN activation alone is sufficient for aversive associations with odors. The population of DANs that can replace the US overlaps with the population of DANs required for BGAM. Collectively, the blockade of MBON‐γ1pedc allows DANs to replace the aversive US to make the aversive associations.

The article "Suppression of a single pair of mushroom body output neurons in Drosophila triggers aversive associations" was published in 2017. Journal: FEBS Open Bio.

Assuming that BGAM is acquired by MBON‐γ1pedc and DANs, there are two questions about the BGAM formation. One is about the pathway for MBON‐γ1pedc to modify DANs effects and the other is about the trigger for DANs activation. The pathway for MBON‐γ1pedc to modify the DANs is unknown although there is anatomical connectivity. According to the previous study referring to the anatomies of MBONs and DANs, the dendrites of a few DANs are slightly co‐localized with the axons of MBON‐γ1pedc 9. This indicates that some DANs may be downstream of MBON‐γ1pedc at the level of a neural circuit. However, we could not detect the functional connectivity of MBON‐γ1pedc and DANs, since the DANs activity was stochastic and fluctuated at the restrictive temperature used to manipulate the MBON‐γ1pedc in the functional calcium imaging (data not shown). Thus, other methodologies, such as optogenetics, membrane potential indicators or synaptic output indicators might be useful to test this possibility. Since MBON‐γ1pedc axons and DANs dendrites are only slightly colocalized, this possibility is less likely than the following second possibility. Second possibility is that MBON‐γ1pedc affects DANs effect indirectly. MBON‐γ1pedc axons are projected to the crepine (a region surrounding the horizontal and medial lobes) and the core of the α and β lobes 9, and the DANs axons also project to the α and β lobes 9, 42. Thus, DANs and MBON‐γ1pedc converge on the lobes, and they may input to KCs or other MBONs coordinately, to modulate their plasticity. Since MBON‐γ1pedc is GABAergic, MBON‐γ1pedc may inhibit the KCs activity, and blocking MBON‐γ1pedc may disinhibit the KCs activity, leading to the hyperactivity of KCs and the easy association with weak DANs activity.

It is also unclear why and how the DANs are activated when MBON‐γ1pedc is blocked and the odors are presented. One possibility is that DANs activity fluctuates, reflecting inner physiological states 27, 28, and that the active state of DANs can stochastically cause aversive memory to a given odor. Another possibility is that the exposure to a given odor activates DANs. We examined the activity of DANs via functional calcium imaging under a two‐photon microscope, but we only observed stochastic activity of DANs and failed to detect significant correlation with the exposure to odors (data not shown).

The article "Suppression of a single pair of mushroom body output neurons in Drosophila triggers aversive associations" was published in 2017. Journal: FEBS Open Bio.

Without the appropriate activity of MBON‐γ1pedc, the probability of aversive associations might be increased even if the environment contains few aversive stimuli. Although aversive associations are important for animals' survival, an appropriate threshold for memory acquisition is necessary to conserve the energy required to acquire an aberrant memory and to highlight the importance of essential memories. MBON‐γ1pedc might have such a gating function by antagonizing the activity of DANs.

BGAM is acquired by odor presentation and the blockade of MBON‐γ1pedc. MBON‐γ1pedc responds to odors robustly, but its response is decreased after associating the odors with ESs or activation of DANs 26, 30. Thus, BGAM acquisition may mimic the situation in which flies sense CS+ odors after associating the odors with ESs. After the classical conditioning, CS+ odor presentation may cause some BGAM in flies.

BGAM was observed as behavioral plasticity, and can be categorized into associative or nonassociative memory, depending on the viewpoint. Since BGAM is acquired solely by an odor presentation, BGAM may be categorized as a nonassociative memory or a particular sensitization. In the T‐maze machine, naïve flies avoid odors (MCH or OCT) as compared to the air (this is called odor avoidance), indicating that odors are aversive stimuli for flies to some extent. In wild‐type flies, odorant information may be processed as aversive information, but not stored as aversive memory by inhibiting the memory acquisition processes. However, the blockade of MBON‐γ1pedc may disturb the inhibiting processes, and thus the odorant information may be stored as an aversive memory. A previous study showed that odor avoidance was enhanced by blocking MBON‐γ1pedc 26, and this study indicated that enhanced odor avoidance lasts as memory by blocking MBON‐γ1pedc. The enhancement of responses to pre‐exposed stimuli is called sensitization. In *Drosophila*, behavioral sensitization to odors or neural sensitization to odors around the KCs was not observed, although odor sensitization in sensory neurons was reported 44. In contrast, in *Caenorhabditis elegans*, it was previously reported that behavioral sensitization to odors was regulated by dopamine release to an interneuron 45. This sensitization mechanism in *C. elegans* might be similar to the BGAM mechanism, since their behavioral protocols are nonassociative learning and dopamine‐related. BGAM might be nonassociative memory and lasting sensitization, and in wild‐type flies, MBON‐γ1pedc might suppress the sensitization.

The article "Suppression of a single pair of mushroom body output neurons in Drosophila triggers aversive associations" was published in 2017. Journal: FEBS Open Bio.

However, if BGAM is acquired by associating an odor with a temperature stimulus or another aversive stimulus surrounding the flies, then BGAM may be categorized as associative memory. In order to block synaptic output by using Shi^ts^, the flies are kept at a restrictive temperature (33 °C), which could be an aversive stimulus 37. Although the temperature we used might be slightly aversive for flies, the temperature shifting to 33 °C for 1 min was lower and shorter than the 34 °C shift for 2 min used in a previous study 37, and our protocol was apparently insufficient for the control strains to acquire strong aversive memory (Fig. 3B). If the blockade of MBON‐γ1pedc lowers the threshold for the temperature as the US, then BGAM could result from the association between the odors and the high temperature. In rats, the aversive US pathway is reportedly inhibited by feedback circuits to calibrate the strength of learning after aversive memory formation 46. MBON‐γ1pedc and DANs may comprise a similar circuit in *Drosophila*. To investigate whether aversive information is associated with odor in BGAM, other novel methodologies to block the synaptic output in a freely moving fly in a precise time window without aversive stimuli, such as temperature shifting, are needed.

Taken together, the blockade of MBON‐γ1pedc during odor presentation without US influences the DANs effects directly or indirectly and forms BGAM. We found the novel function of MBON‐γ1pedc for BGAM formation at the level of behavior. The MBON‐γ1pedc functions to suppress the memory formation, indicating that memory acquisition can be regulated negatively. Only a few studies have reported the negative regulation (suppression) of memory, and a recent study reported that the neural circuit suppresses the US pathway in rats by feedback circuits, to calibrate the strength of learning after aversive memory formation 46. This is the first evidence that MBON‐γ1pedc and DANs may comprise a similar circuit in *Drosophila*.

## Author contributions

YU, MH and TT conceived and designed the project. YU acquired the data. YU, MH, TA and TT analyzed and interpreted the data. YU and TT wrote the paper.
